# Effect of Controlled Microtopography on Osteogenic Differentiation of Mesenchymal Stem Cells

**DOI:** 10.1155/2022/7179723

**Published:** 2022-01-28

**Authors:** Chengxin Chen, Yuanjing Zhu, Ran Wang, Yu Han, Hongbo Zhou

**Affiliations:** Xiangya Stomatological Hospital and Xiangya School of Stomatology, Central South University, Changsha, Hunan 410008, China

## Abstract

Various kinds of controlled microtopographies can promote osteogenic differentiation of mesenchymal stem cells (MSCs), such as microgrooves, micropillars, and micropits. However, the optimal shape, size, and mechanism remain unclear. In this review, we summarize the relationship between the parameters of different microtopographies and the behavior of MSCs. Then, we try to reveal the potential mechanism between them. The results showed that the microgrooves with a width of 4–60 *μ*m and ridge width <10 *μ*m, micropillars with parameters less than 10 *μ*m, and square micropits had the full potential to promote osteogenic differentiation of MSCs, while the micromorphology of the same size could induce larger focal adhesions (FAs), well-organized cytoskeleton, and superior cell areas. Therefore, such events are possibly mediated by microtopography-induced mechanotransduction pathways.

## 1. Introduction

Surface topography have effects on cellular responses including contact guidance and influence on cellular functions, which have been proven for several years [1, 2]. Recently, due to the advances in microfabrication technologies and the tremendous flexibility in shape and size of topographical features [3], the study interest in exploring microtopographical cues for inducing bone regeneration has substantially accelerated. Generally, microtopographies can be designed to affect the relevant cells by mimicking the native extracellular matrix (ECM) of them. While microtopography at scale above 100 *μ*m mainly influence cells at colony level, microscale between 0.1 and 100 *μ*m affects cells at the single level [4].

Dental implantation in partial or totally edentulous patients is a predictable treatment with high rates of long-term success [5]. However, early osseointegration is still considered a challenge in areas with the most trabeculated bone (bone type IV) together with lower-density and thinner cortical bone, which is generally considered less suitable for supporting dental implants [6]. Mesenchymal stem cells (MSCs) are among the earliest cells to colonize on the implant surface after placement, which are the precursors to bone forming osteoblasts [7, 8]. In recent years, implant surface with microscale designs such as microgrooves [9–11], micropillars [12, 13], and micropits [14, 15] have been created to induce the osteogenic differentiation behavior of MSCs and improve the osseointegration, allowing immediate or early functional loading in patients with reduced bone density. Therefore, inducing the differentiation of MSCs towards the osteoblast lineage by providing microtopographical cues may assist more rapid and stable osseointegration. Although micropatterns can enhance osteogenic differentiation of MSCs, there is no consensus on the optimal scale and the mechanism is still unknown.

In this review, we have the unique intention of summarizing the presently available experimental evidence to investigate the relation between microtopographic parameters and MSC differentiation. Then, we attempt to identify the potential mechanism with regard to how microtopographies affect manual osteogenic differentiation of MSCs in vitro. We hope these will provide reference for future implant surface topography design.

## 2. Microfabrication Technologies

With microfabrication technology, it is possible to operate on microtopographies for controlling or inducing stem cell differentiation. Currently, technologies for fabrication of microtopographies include direct fabrication methods, involving photolithography [16] and laser photoablation [17]; and indirect (prototyping) techniques, such as hot embossing [18] and soft lithography [19].  Table 1 presents the advantages and disadvantages of these technologies.

### 2.1. Laser Photoablation

Femtosecond laser micromachining (Figure 1(a)) has been efficiently carried out to supply micropatterns in titanium and zirconia [15, 20, 21]. The laser pulses travelled through air to the focusing device, which can focus the beam and position the sample. Samples were located on a motorised platform with three-axis motion, in order that pulses can impinge perpendicularly onto their surfaces [22, 23].

### 2.2. Photolithography

Micropatterns in titanium and silicon have been generated by photolithography [16, 24], producing the patterning of a layer of photosensitive polymer (photoresist) by utilizing UV (Figure 1(b)) or X-ray light (Figure 1(c)). The light is shone through a “mask” containing the designed pattern in the form of UV-opaque features on a UV-transparent background [25]. Then, the pattern can be transferred to the substrate by the next dry (e.g., ICP-based dry etching) or wet etching (e.g., hydrofluoric acid)[26, 27].

### 2.3. Hot Embossing

Hot embossing (Figure 2(a)) has been used to produce polystyrene microgroove surfaces [29]. In hot embossing imprint lithography, a micromachined master (typically of silicon) is pressed right into a thermoplastic fabric at an elevated temperature and it forms relief patterns in the polymer. The major advantages of this technology include its low cost and the ability to generate 3D features, which are very difficult to produce in silicon for other technologies [18].

### 2.4. Soft Lithography

Microgrooves, micropits, and micropillars have been, respectively, produced by soft lithography (Figure 2(b)) on a polymer [12, 14, 30]. Soft lithography is an ensemble of techniques that collectively employ elastomeric polymers, which are primarily based on polydimethylsiloxane (PDMS)—within the form of a mold, stamp, or mask because of the critical element of a pattern-forming method [31].

## 3. Physical Properties of Micropatterns

Surface roughness and wettability are two important physical properties of micropatterns, which may contribute to osteogenic differentiation of MSCs. Surface roughness altered the adhesion state and geometric shape of cells [32, 33]. The cytoskeleton of MSCs showed higher tension on the rougher surface by sensing the roughness gradient, which was further transferred to the nucleus and finally affected the expression of osteogenic markers of stem cells. Meanwhile, it is founded that MSCs on the surface with moderate wettability presented a higher level of gene expression of integrin than those on the more hydrophobic surfaces [34]. It is well known that integrin receptors mediate cell-matrix interactions and play a central role in cell adhesion, spreading, migration, proliferation, and osteogenic differentiation [35, 36]. Therefore, surface wettability can influence osteogenic differentiation of MSCs via integrin.

### 3.1. Microgroove

The microgrooves are composed of grooves and ridges, arranged in a line (Figure 3). Because they can be relatively easily fabricated with various microfabrication techniques, such as photolithography [37], laser photoablation [38], and so on, they have been extensively investigated for their effects on cell behavior. The influence of the microgroove on the surface wettability has been reported, which exhibited the lower contact angles compared to the untreated ones [20]. On the contrary, the textured surfaces of zirconia showed higher contact angles [39]. This difference may be due to the different material substrates used.

### 3.2. Micropillar

Micropillar is one-dimensional shape perpendicular to the substrate surface (Figure 4), which is also usually followed to observe interaction between cell and material. On polymer and SiO_2_ films, micropillars of different heights, side lengths, and gap sizes can be fabricated by soft lithography and sol-gel methods [12, 40]. The contact angle increased appreciably within the presence of the patterned features, with the pillar array surface supplying a hydrophilic behavior while the line array thin film presented relatively high hydrophobicity values [40].

### 3.3. Micropit

These micropit substrates comprise arrays of square or round shapes (Figure 5). Side length (diameter) and depth are the two main parameters of micropits. At present, soft etching and femtosecond laser can be used to fabricate micropits of different scales in polymers [14] and zirconia [15], respectively. However, the physical properties of the micropit surface, such as hydrophilicity need to be further studied.

## 4. Regulation of Micropatterns on Cell Adhesion and Morphology

Micropatterns provide a wide opportunity for the fabrication of surface with defined shape, size, and spatial arrangement. This permits researchers to explore the interactions between micropatterns and MSCs, including cellular adhesion, morphology, and osteogenic differentiation. Investigation of these interactions may additionally display capability molecular mechanisms concerned in MSCs alterations in osteogenic differentiation to micropatterns.

### 4.1. Microgroove

For microgrooved topographies, it allowed cellular attachment after 24 hours and the cell morphology was dependent on the topographical cue [21, 29]. The cells were aligned in the path parallel to the grooves with cytoskeleton clearly elongating. While on the unpatterned surface, cells were orientated randomly and presented a spread phenotype with distinct cytoplasmic processes. Additionally, it reported that the focal adhesions (FAs) were less, smaller, and oriented in several directions on the untreated samples. On the contrary, cells adhesion to the microtopography was much stronger and oriented according to the microfeatures, displaying very mature FAs. Further research also found that [10] microgrooves with various widths prompted differential expression of diverse genes including cellular adhesion, migration, and cytoskeletal reorganization. Considering that the topographical feature could modulate cell adhesion signaling and cytoskeletal organization, four essential FA-related protein expression were investigated involved in integrin *β*1, integrin *α*5, vinculin, and talin [9]. The outcomes indicated that the expression of integrin *β*1 and *α*5 is substantially upregulated on the microgroove surface compared with the flat one.

### 4.2. Micropillar

It was reported earlier that micropillars could enhance cell attachment [12, 41], which may be due to a larger contact area and maturation of FAs assisted by space patterns.

The research of MSCs cultured on micropillars with different heights has found that feature height influences FA size and density [42]. After 24-hour attachment, mature FAs were observed on the height of 0.8 *μ*m micropillar and flat one. When the micropillar height increases to 4.6 *μ*m or larger, FAs were densely distributed around the micropillars. Recently, it reported that a substantially higher number of MSCs attached on the modified surfaces in comparison with the flat one presented a positive regulation of micropillars on cell attachment [12]. While the number of attached cells was also found to be affected by pillar side length (P) and interpillar gap size (G). Compared with other sizes, cell attachment was better on P4G4. Given that the edges of pillar tops had been proven to be the place where focal contacts were primarily targeting [43], cell attachment better on P4G4 become possibly the consequence of the highest number of pillars per unit area that cells can interact. As for cellular morphology, they were squeezed and conformed cytoplasm to the interpillar spaces, which constrains their typical spread morphology attachment on the flat control [12, 40].

### 4.3. Micropit/Microwell

In order to evaluate the effect of micropits surfaces on FA enhancement, the immunostaining was performed at day 2, which indicated that the FAs were matured inside the pits and distributed around the peripheral of the cells [14]. While the matured FA areas were significantly larger on the micropit surfaces than that on the control surface. The cell shape of MSCs cultured on micropits of different depths and diameters has shown that cell morphology varied relying on the pattern type. Stanciuc et al. [15]. indicated that when the diameter was 30 *μ*m, higher depth contributed to higher proportion of polygonal cells and larger cell area. If cells cultured on areas with smaller dimensions, especially on the regions with the diameter of 10 *μ*m and depth of 3 or 10 *μ*m, it had a more elongated cell morphology. Talking about the cell position, MSCs were preferentially distributed inside the microwells, especially at the early culture stage when the cell confluence was at a low level [44]. Although the mechanism of this difference still needs to figure out, it may be due to the various spatial situation of physical and biochemical signals inside and outside the micropits.

The abovementioned results indicated that micropatterns could influence MSCs adhesion by mediating FA size, density, and altering integrin expression. Micropatterns with appropriate size and space arrangement may offer the essential physical cues that cell receptors require to regulate cell morphology, reorganize the cytoskeleton, and transmit mechanical signals towards the nucleus, which may ultimately contribute to alterations in stem cell differentiation.

## 5. Regulation of Micropatterns on Osteogenic Differentiation

In vivo, surface roughness of the dental implant is essential for the integration in tissue regeneration or tissue engineering [45, 46]. Also, some studies have confirmed it was able to have an effect on the expression of osteogenic markers of stem cells [47, 48]. However, the surface roughness is difficult to be characterized. Instead, the substrates with ordered surface topographies are relatively simple to characterize while increasing roughness, such as microgroove, micropillar, and micropit.

As mentioned in the previous segment, the ordered surface topographies could induce large FAs, an organized cytoskeleton, and a well-spread morphology of MSCs. According to the report, large spreading and increased contractility of MSCs prefer osteogenic differentiation, while small cell spreading and low contractility prefer adipogenic differentiation [49]. Therefore, the specific microtopographies feature could induce the osteogenic differentiation of MSCs as well as regulate the cell adhesion and morphology.

### 5.1. Microgroove

The groove and ridge width are two important parameters to regulate cell osteogenic differentiation, and the experimental details of several research studies are presented in Table 2.

The groove width of 4 *μ*m and ridge width of 2 *μ*m tended to promote osteogenic differentiation when the Ad-MSCs (adipose-derived mesenchymal stem cells) were seeded on the substrate [11]. Then, it was reported that a specific microgroove with a groove width of 7 *μ*m and ridge width of 3 *μ*m can most effectively induce osteogenic differentiation of mMSCs (mouse bone marrow-derived mesenchymal stem cells) [9]. At the same time, the surface feature showed the highest level of protein expression of integrin, which is an important component of FAs. This indicated that there is a connection between cell adhesion and osteogenic differentiation of MSCs. Abagnale et al.[50] systematically varied the width of grooves and ridges, ranging from 2 to 15 *μ*m. Notably, there was a gradual reduction of osteogenic differentiation with increasing ridge width. On the 15 *μ*m ridges hMSCs (human bone marrow-derived mesenchymal stem cells) revealed consistently higher adipogenic differentiation rather than osteogenic differentiation. When the groove width is increased to be 30 or 60 *μ*m, the researcher found it could also significantly enhance the osteogenic differentiation of hMSCs [10], while the groove width of 60 *μ*m would show a peak in the difference of osteogenic differentiation (signaled by extracellular calcium deposition) on day 21 [51]. When the groove width achieves>100 *μ*m, the ALP activity level of hMSCs was increased slightly on day 7, but no statistical difference became determined on day 14 [52]. These results reveal that the micropattern with groove width of about 4–60 *μ*m and ridge width of <10 *μ*m is probably suitable for osteogenic differentiation of MSCs.

### 5.2. Micropillar

It is an effective way to apply micropillar with fine-tuned dimensions to enhance osteogenic performance in vitro and in vivo, which can imitate 3D characteristics of the bone microstructure on material surfaces.  Table 3 shows the main results of some studies.

The effect of different heights of micropillar on MSCs osteogenic differentiation in vivo has been revealed. It indicated that on the 5 *μ*m-high pillar, rMSCs(rat bone marrow-derived mesenchymal stem cells) still have the ability of osteogenic differentiation although their nuclei were severely deformed [53]. In order to further explore the impact of micropillar height on the osteogenic performance of MSCs, several studies reported that the micropillar height of 3 *μ*m or 6.4 *μ*m promoted osteogenic differentiation, while the lower height of 0.8 *μ*m enhanced adipogenic performance [40, 42]. Konttinen [54] found that square micropillar with the height of 5 *μ*m might be better for osteogenic differentiation of MSCs in comparison to the height of 0.2 *μ*m or 20 *μ*m. In addition to the height, the side length of the square micropillar (P) and the interpillar gap(G) are also crucial factors for cell osteogenic differentiation. Using photolithography, three types of square micropillar were created with the height of 8 *μ*m. The results indicated that hydrophobic micropillar, which is with lateral dimensions of 4 *μ*m (P4G4) and 8 *μ*m (P8G8), respectively, induced mineralization in bone nodule-like cell aggregates and the expression of early osteogenic genes without any differentiation supplements in the growth media [12]. It can be worth noting that the micropillar structure may be more conducive to osteogenic differentiation, when the three parameters are within 10 *μ*m.

### 5.3. Micropit

The micropit structures have certified their importance in modulating the behavior of pluripotent stem cells. For example, they have been proved to induce the growth of stem cells and can promote them to generate homogeneous cell colonies, which are with defined shapes and sizes. However, there is confined information at the effect of micropit geometry on the osteogenic differentiation of MSCs.

The micropits were created in two different shapes: square and round [55]. They were produced by soft lithography, with different lengths or diameters and an identical depth of 10 *μ*m. It was found that the square micropits surface with 50 *μ*m side length induces the proliferation and osteogenic performance of MSCs compared to the round-shaped micropits substrate with 50 *μ*m diameter. Seo et al. [14] also used soft lithography to produce micropits with 3 *μ*m side length, 2 *μ*m or 4 *μ*m depth on PDMS. Compared to the control flat surfaces, the activity of ALP was significantly higher on the micropit surfaces at day 7 and the intensity of OCN protein followed similar trends with ALP. However, pits with 30 *μ*m diameter and 10 *μ*m deep might induce MSCs commitment towards the osteoblastic phenotype in contrast to unpatterned or feature surface with smaller size, such as 10 and 20 *μ*m diameter [15]. These mentioned studies discovered that the square-shaped micropit with large side length may be better for osteogenic performance of MSCs. As for round microstructure, it needs more systematic investigation. The research details are summarized in Table 4.

In general, the abovementioned consequences have presented more sensitivity of osteogenic performance of MSCs to feature size when cultured on micropatterns. Moreover, it appears to be a connection between the cell adhesion and osteogenic differentiation of MSCs seeded on micropatterns. As it was mentioned before, the identical size can effectively induce large FAs, a well-organized cytoskeleton, and a typical spread morphology of MSCs. To further analyse this connection, potential mechanotransduction mechanisms need to be investigated, which require FAs to transduct signals from the extracellular matrix (ECM) to the cell through integrin and intracellular protein-cytoskeleton complex.

## 6. Potential Mechanisms Concerned in Microtopography-Induced Osteogenic Differentiation

Mechanical signals are converted intracellularly into biochemical signals which are induced by surface topography through a process called mechanotransduction [56, 57]. So far, the results in vitro indicated that the mechanotransduction involved in the microtopography-induced osteogenic performance [13, 58, 59]. There are two kinds of mechanisms of mechanotransduction that can be listed as follows, which may concern with integrin signaling, cytoskeleton reorganizing, and nuclear mechanotransduction. One way is named direct mechanotransduction. Its content is that the stress or mechanical force of microtopography propagates into the nucleus through the cytoskeleton to regulate nucleus form and probably chromosome orientation directly. The second mechanism is indirect mechanotransduction. It means that mechanical signals convert into biochemical signals via biomolecules.

The direct physical mechanotransduction (Figure 6) is essential for transferring mechanical cues of the microtopographical surface into the nucleus, including exertion of stress from the cytoskeleton on the nucleoskeleton. Nuclear organization is hierarchical, consisting of chromosome territories. The microtopography-induced signals can be transported into the nucleus directly via cytoskeleton elements acting as an integrated unit. The experimental results indicating chromosomal repositioning and nucleus deformation in reaction to microtopography suggest that the nucleus can be regarded as a positive mechanosensor [60]. This is backed up by nuclear lamina, which can provide structural support to the nucleus and form the link to the actin cytoskeleton, guaranteeing the appropriate nuclear and centrosomal organization [61]. By this means, the stress can be directly conveyed from the actin cytoskeleton to the nuclear and chromosomes with feasible subsequent consequences on gene expression [9, 62]. MSCs possess an actin cytoskeleton and have been shown to remodel in response to microtopography. This remodelling instigates subsequent mechanotransductive pathways, ultimately leading to the more expression of osteogenic genes such as RUNX-2, OPN, and so on. Application of a stretching force to MSCs generating strain also increases their proliferation and the production of the bone matrix protein. The abovementioned findings suggest the vital role of direct mechanotransduction in cellular response to microtopography. However, the connection between the mechanotransduction mechanisms and specific micropatterns features still needs to be further investigated.

Next to the direct mechanotransductive signaling pathways, it reported that RhoA-ROCK-MLCK (myosin II) is a distinct indirect pathway [46] (Figure 7). RhoA, acting as a mechanotransduction receptor, plays a distinctive role in regulating actin cytoskeletal reorganization [64]. Activating the downstream of RhoA/ROCK pathway will increase the polymerization of the cytoskeleton by the way of formation of large c and stress fibers. This mechanism is supported by molecular researches indicating that higher RhoA activity is connected with enhanced adhesion maturation, cellular stress, and cytoskeleton reorganizing that promote osteogenic performance of MSCs [43, 65]. Their role has been additionally confirmed by the use of small molecular inhibitors, blebbistatin and Y-27632, to inhibit myosin II and ROCK, respectively. It determined that the FA formation, cytoskeleton reorganizing, and FAKs (focal adhesion kinases) phosphorylation were dramatically reduced. At the same time, the topographical dependency of FA formation was also fantastically decreased. Following mechanical stimulation of integrins by external microtopography, the extensive FAs with other kinases, including FAKs and extracellular signal-related kinases (ERKs) [66], bring about force concentration of actin. Finally, the nuclear deformation causing by force upregulates the expression of RUNX2 and OPN gene in MSCs, further demonstrating the importance of signal transduction pathways in altering cell responses to mechanical stimuli. These findings indicate that signal transduction pathways can regulate the adhesion and cytoskeleton organization of MSCs on the microtopography [43], which may finally affect the expression of osteogenic genes.

## 7. Conclusions and Outlook

To apprehend the connections between microtopographies and cellular activities, different types of patterns (groove, pit, and pillar) have been developed. Here, we review fabrication methods for acquiring physically patterned microscale surfaces and discuss physical properties of patterns. Then, we focus on the relationships between MSCs responses and microtopogracial feature, which could be carried out to modify dental implant surface. The preference for large FAs on microtopographical surface suggests that osteogenic performance and cellular adhesion are associated. In addition, a well-spread morphology with a highly organized cytoskeleton will be beneficial for osteogenic differentiation, indicating that direct mechanotransduction mechanism ought to play an important role in the connection between MSCs adhesion behavior and osteogenic performance. Although controlled microtopography can be regarded as a potential cue for guiding MSCs differentiation towards the osteoblast lineage, no optimal micropatterns have been confirmed yet. Also, the reason for that is a lack of systematic comparison of the outcomes of various micropattern dimensions and spatial arrangements. Next, we need to further improve the microfabrication processes for biomedical materials and study the underlying mechanisms of interaction between micropatterns and MSCs to screen the optimal micropattern structure and size.

## Figures and Tables

**Figure 1:** Illustrations of the direct fabrication techniques: (a) laser micromachining, (b) photolithography,.and (c) X-ray lithography. Images (a)–(c) were reprinted from [28].

**Figure 2:** Illustrations of the prototyping techniques: (a) hot embossing and (b) soft lithography. Images (a-b) were reprinted from [28].

**Figure 3:** Structure of the microgroove substrate.

**Figure 4:** Structure of the micropillar substrate.

**Figure 5:** Structure of the micropit substrate.

**Figure 6:** Schematics showing the mechanism of direct physical mechanotransduction. Microtopography induced cell focal adhesion maturation and actin organization with enhanced contraction force.

**Figure 7:** Schematics showing the mechanism of indirect pathway. This process involved integrin recruitment and phosphorylation of focal adhesion kinase (FAK) via the RhoA-ROCK pathway and myosin II.

**Table 1:** The summary of microfabrication techniques.

Methods	Microtopography	Advantages	Disadvantages
Photolithography	Microgroove	Ideal for microstructure	Usually requires a flat surface to start with and chemical post-treatment needed
Laser photoablation	Microgroove and micropit	Wide applicability, high resolution, rapid, repeatable, and contactless process	Multiple treatment sessions and limited
Hot embossing	Microgroove	Cost-effective, precise, rapid, and mass production	Restricted to thermoplastics and difficult to fabricate complex 3D structures
Soft lithography	Microgroove, micropit, and micropillar	Cost-effective and able to fabricate 3D geometries high resolution	Pattern deformation and vulnerable to defect materials

**Table 2:** Summary of MSC differentiation regulated by microgroove.

Material	Groove (*μ*m)	Ridge width (*μ*m)	Depth (*μ*m)	Cell type	Main results
PDMS	0.65–6	0.35–7	0.1–2	Ad-MSCs	Groove width of 4 *μ*m and ridge width of 2 *μ*m promotes osteogenic differentiation greatly
Ti	7–20	3–20	2	mMSCs	Groove width of 7 *μ*m and ridge width of 3 *μ*m can most effectively align the cells and promote osteogenic differentiation
Polyimide	2–15	2–15	5	hMSCs	Groove width of 10 *μ*m and ridge width of 10 *μ*m can promote osteogenic differentiation whereas 15 *μ*m ridges supports adipogenic differentiation
Ti	30 and 60	—	10	hMSCs	Groove width of 30 or 60 *μ*m enhances osteogenic differentiation
Ti	60	—	10 and 20	hMSCs	Groove width of 60 *μ*m and depth of 10 *μ*m allows for the highest levels of adhesion and osteogenic differentiation on day 21
PCL	50, 100, and 200	—	25, 50, and 100	hMSCs	Groove width >100 *μ*m slightly increases the ALP activity level of MSCs.

PDMS, polydimethylsiloxane; Ti, titanium; PCL, polycaprolactone.

**Table 3:** Summary of MSC differentiation regulated by micropillar.

Material	Height (*μ*m)	Side length (*μ*m)	Gap size	Cell type	Main results
PLGA	0.2, 1, and 5	3–6	6	rMSCs	rMSCs are able to enhance osteogenic differentiation, despite the nuclei of cells are severely deformed on micropillars of 5 *μ*m height
SiO2	3	5	10	hMSCs	The height of 3 *μ*m of microtopographic features could promote osteogenic differentiation
PLGA	0.8, 3.2, 4.6, 5.3, and 6.4	3	—	rMSCs	The height of 4.6 or 6.4 *μ*m promotes osteogenic differentiation.
Hybrid polymer	0.2, 5, and 20	100	100	hMSCs	Lower pillar promotes osteogenic differentiation
PMMA	8	4,8,16	4,8,16	DPSCs	Micropillar arrays with lateral dimensions of 4 *μ*m (P4G4) and 8 *μ*m (P8G8) induce the expression of early osteogenic genes

PLGA, poly(d,l-lactide-co-glycolide); PMMA, poly(methyl methacrylate); DPSCs, human dental pulp stem cells.

**Table 4:** Summary of MSC differentiation regulated by micropit.

Material	Shape	Depth (*μ*m)	Side length /diameter (*μ*m)	Cell type	Main results
PS	Square and round	10	10, 25, and 50	Ad-MSCs	Square micropit with a side length of 50 *μ*m shows advantages over round-shaped micropits
PDMS	Square	2 and4	3	mMSCs	Cells on the substrates has enhanced FAs, actin polymerization, and osteogenic differentiation
Zirconia	Round	3 and 10	10, 20, and 30	hMSCs	Pits with 30 *μ*m diameter and 10 *μ*m deep may significantly promote MSCs commitment towards the osteoblastic phenotype

PS, polystyrene.

## Data Availability

The data used to support the findings of this study are included within the review.

## References

[1] Walboomers X. F., Croes H. J. E., Ginsel L. A., Jansen J. A. (1998). Growth behavior of fibroblasts on microgrooved polystyrene. *Biomaterials*.

[2] Lee S. J., Choi J. S., Park K. S., Khang G., Lee Y. M., Lee H. B. (2004). Response of MG63 osteoblast-like cells onto polycarbonate membrane surfaces with different micropore sizes. *Biomaterials*.

[3] Grenci G., Bertocchi C., Ravasio A. (2019). Integrating microfabrication into biological investigations: The benefits of interdisciplinarity. *Micromachines*.

[4] Dalby M. J., Gadegaard N., Oreffo R. O. C. (2014). Harnessing nanotopography and integrin-matrix interactions to influence stem cell fate. *Nature Materials*.

[5] Frisch E., Wild V., Ratka‐Krüger P., Vach K., Sennhenn‐Kirchner S. (2020). Long‐term results of implants and i mplant‐supported prostheses under systematic supportive implant therapy: a retrospective 25‐year study. *Clinical Implant Dentistry and Related Research*.

[6] Sakka S., Baroudi K., Nassani M. Z. (2012). Factors associated with early and late failure of dental implants. *Journal of Investigative and Clinical Dentistry*.

[7] Caplan A. (2009). Why are MSCs therapeutic? New data: New insight. *The Journal of Pathology*.

[8] Azizeh-Mitra Y., James P. F., Rosa A., Aswati S., Conor F., Hassane O. (2016). Prospect of stem cells in bone tissue engineering: a review. *Stem Cells International*.

[9] Zhu M., Ye H., Fang J. (2019). Engineering high-resolution micropatterns directly onto titanium with optimized contact guidance to promote osteogenic differentiation and bone regeneration. *ACS Applied Materials & Interfaces*.

[10] Lee M. H., Kang J. H., Lee S. W. (2012). The significance of differential expression of genes and proteins in human primary cells caused by microgrooved biomaterial substrata. *Biomaterials*.

[11] Kim C.-S., Kim J.-H., Kim B., Park Y.-S., Kim H.-K., Hieu Trung T. (2017). A specific groove pattern can effectively induce osteoblast differentiation. *Advanced Functional Materials*.

[12] Hasturk O., Ermis M., Demirci U., Hasirci N., Hasirci V. (2019). Square prism micropillars on poly(methyl methacrylate) surfaces modulate the morphology and differentiation of human dental pulp mesenchymal stem cells. *Colloids and Surfaces B: Biointerfaces*.

[13] Zanchetta E., Guidi E., Della Giustina G. (2015). Injection molded polymeric micropatterns for bone regeneration study. *ACS Applied Materials & Interfaces*.

[14] Seo C. H., Jeong H., Feng Y. (2014). Micropit surfaces designed for accelerating osteogenic differentiation of murine mesenchymal stem cells via enhancing focal adhesion and actin polymerization. *Biomaterials*.

[15] Stanciuc A.-M., Flamant Q., Sprecher C. M., Alini M., Anglada M., Peroglio M. (2018). Femtosecond laser multi-patterning of zirconia for screening of cell-surface interactions. *Journal of the European Ceramic Society*.

[16] Ponomarev V. A., Shvindina N. V., Permyakova E. S. (2019). Structure and antibacterial properties of Ag-doped micropattern surfaces produced by photolithography method. *Colloids and Surfaces B: Biointerfaces*.

[17] Schieber R., Lasserre F., Hans M. (2017). Direct laser interference patterning of CoCr alloy surfaces to control endothelial cell and platelet response for cardiovascular applications. *Advanced Healthcare Materials*.

[18] Charest J. L., Bryant L. E., Garcia A. J., King W. P. (2004). Hot embossing for micropatterned cell substrates. *Biomaterials*.

[19] Weibel D. B., Diluzio W. R., Whitesides G. M. (2007). Microfabrication meets microbiology. *Nature Reviews Microbiology*.

[20] Wang C., Hu H., Li Z. (2019). Enhanced osseointegration of titanium alloy implants with laser microgrooved surfaces and graphene oxide coating. *ACS Applied Materials & Interfaces*.

[21] Carvalho A., Cangueiro L., Oliveria V., Vilar R., Fernandes M. H., Monteiro F. J. (2018). Femtosecond laser microstructured Alumina toughened Zirconia A new strategy to improve osteogenic differentiation of hMSCs. *Applied Surface Science*.

[22] Martínez-Calderon M., Manso-Silván M., Rodríguez A. (2016). Surface micro- and nano-texturing of stainless steel by femtosecond laser for the control of cell migration. *Scientific Reports*.

[23] Luo F., Wang L., Xiao Z. (2021). Application of femtosecond laser microfabrication in the preparation of advanced bioactive titanium surfaces. *Journal of Materials Chemistry B*.

[24] Kim E.-C., Lee D. Y., Lee M.-H. (2018). The effect of fibronectin-immobilized microgrooved titanium substrata on cell proliferation and expression of genes and proteins in human gingival fibroblasts. *Tissue Engineering and Regenerative Medicine*.

[25] Kang M., Byun J. H., Na S., Jeon N. L. (2017). Fabrication of functional 3D multi-level microstructures on transparent substrates by one step back-side UV photolithography. *RSC Advances*.

[26] Parker E. R., Thibeault B. J., Aimi M. F., Rao M. P., MacDonald N. C. (2005). Inductively coupled plasma etching of bulk titanium for MEMS applications. *Journal of the Electrochemical Society*.

[27] Kim H.-J., Lee S.-H., Lee J. (2015). Controlled patterning of vertical silicon structures using polymer lithography and wet chemical etching. *Journal of Nanoscience and Nanotechnology*.

[28] Wu J., Gu M. (2011). Microfluidic sensing: State of the art fabrication and detection techniques. *Journal of Biomedical Optics*.

[29] Sun L., Pereira D., Wang Q. (2016). Controlling growth and osteogenic differentiation of osteoblasts on microgrooved polystyrene surfaces. *PLoS One*.

[30] Kwon C., Kim Y., Jeon H. (2017). Collective migration of lens epithelial cell induced by differential microscale groove patterns. *Journal of Functional Biomaterials*.

[31] Qin D., Xia Y., Whitesides G. M. (2010). Soft lithography for micro- and nanoscale patterning. *Nature Protocols*.

[32] Yang W., Han W., He W. (2016). Surface topography of hydroxyapatite promotes osteogenic differentiation of human bone marrow mesenchymal stem cells. *Materials Science and Engineering: C*.

[33] Shahrousvand M., Sadeghi G. M. M., Shahrousvand E., Ghollasi M., Salimi A. (2017). Superficial physicochemical properties of polyurethane biomaterials as osteogenic regulators in human mesenchymal stem cells fates. *Colloids and Surfaces B: Biointerfaces*.

[34] Hao L., Yang H., Du C. (2014). Directing the fate of human and mouse mesenchymal stem cells by hydroxyl-methyl mixed self-assembled monolayers with varying wettability. *Journal of Materials Chemistry B*.

[35] Rosa A. L., Kato R. B., Castro Raucci L. M. S. (2014). Nanotopography drives stem cell fate toward osteoblast differentiation through *α*1*β*1 integrin signaling pathway. *Journal of Cellular Biochemistry*.

[36] Docheva D., Popov C., Mutschler W., Schieker M. (2007). Human mesenchymal stem cells in contact with their environment: Surface characteristics and the integrin system. *Journal of Cellular and Molecular Medicine*.

[37] Ha M., Athirasala A., Tahayeri A., Menezes P. P., Bertassoni L. E. (2020). Micropatterned hydrogels and cell alignment enhance the odontogenic potential of stem cells from apical papilla in-vitro. *Dental Materials*.

[38] Carvalho A., Cangueiro L., Oliveira V., Vilar R., Fernandes M. H., Monteiro F. J. (2018). Femtosecond laser microstructured Alumina toughened Zirconia: A new strategy to improve osteogenic differentiation of hMSCs. *Applied Surface Science*.

[39] Carvalho A., Grenho L., Fernandes M. H. (2019). Femtosecond laser microstructuring of alumina toughened zirconia for surface functionalization of dental implants. *Ceramics International*.

[40] Carvalho A., Pelaez-Vargas A., Hansford D. J., Fernandes M. H., Monteiro F. J. (2016). Effects of line and pillar array microengineered SiO2 thin films on the osteogenic differentiation of human bone marrow-derived mesenchymal stem cells. *Langmuir*.

[41] Hasturk O., Ermis M., Demirci U., Hasirci N., Hasirci V. (2018). Square prism micropillars improve osteogenicity of poly(methyl methacrylate) surfaces. *Journal of Materials Science: Materials in Medicine*.

[42] Liu X., Liu R., Cao B. (2016). Subcellular cell geometry on micropillars regulates stem cell differentiation. *Biomaterials*.

[43] Seo C. H., Furukawa K., Montagne K., Jeong H., Ushida T. (2011). The effect of substrate microtopography on focal adhesion maturation and actin organization via the RhoA/ROCK pathway. *Biomaterials*.

[44] Xu X., Wang W., Kratz K. (2015). Controlling major cellular processes of human mesenchymal stem cells using microwell structures. *Advanced Healthcare Materials*.

[45] Matos G. R. M. (2021). Surface roughness of dental implant and osseointegration. *Journal of Maxillofacial and Oral Surgery*.

[46] Boyan B. D., Lotz E. M., Schwartz Z. (2017). Roughness and hydrophilicity as osteogenic biomimetic surface properties. *Tissue Engineering Part A*.

[47] Hou Y., Yu L., Xie W. (2020). Surface roughness and substrate stiffness synergize to drive cellular mechanoresponse. *Nano Letters*.

[48] Xia J., Yuan Y., Wu H., Huang Y., Weitz D. A. (2020). Decoupling the effects of nanopore size and surface roughness on the attachment, spreading and differentiation of bone marrow-derived stem cells. *Biomaterials*.

[49] Chen G., Kawazoe N., Chun H. J., Reis R. L., Motta A., Khang G. (2020). Regulation of stem cell functions by micro-patterned structures. *Biomimicked Biomaterials: Advances in Tissue Engineering and Regenerative Medicine*.

[50] Abagnale G., Steger M., Nguyen V. H. (2015). Surface topography enhances differentiation of mesenchymal stem cells towards osteogenic and adipogenic lineages. *Biomaterials*.

[51] Leesungbok R., Lee S. W., Ahn S. J. (2012). Specific temporal culturing and microgroove depth influence osteoblast differentiation of human periodontal ligament cells grown on titanium substrata. *Tissue Engineering and Regenerative Medicine*.

[52] Zhang Q., Dong H., Li Y. (2015). Microgrooved polymer substrates promote collective cell migration to accelerate fracture healing in an in vitro model. *ACS Applied Materials & Interfaces*.

[53] Pan Z., Yan C., Peng R., Zhao Y., He Y., Ding J. (2012). Control of cell nucleus shapes via micropillar patterns. *Biomaterials*.

[54] Kaivosoja E., Suvanto P., Barreto G. (2013). Cell adhesion and osteogenic differentiation on three-dimensional pillar surfaces. *Journal of Biomedical Materials Research Part A*.

[55] Xu X., Wang W., Kratz K. (2014). Controlling major cellular processes of human mesenchymal stem cells using microwell structures. *Advanced Healthcare Materials*.

[56] Burridge K., Monaghan-Benson E., Graham D. M. (2019). Mechanotransduction: From the cell surface to the nucleus via RhoA. *Philosophical Transactions of the Royal Society B: Biological Sciences*.

[57] Stewart S., Darwood A., Masouros S., Higgins C., Ramasamy A. (2020). Mechanotransduction in osteogenesis. *Bone & Joint Research*.

[58] Fu J., Liu X., Tan L. (2020). Modulation of the mechanosensing of mesenchymal stem cells by laser-induced patterning for the acceleration of tissue reconstruction through the Wnt/*β*-catenin signaling pathway activation. *Acta Biomaterialia*.

[59] Azeem A., English A., Kumar P. (2015). The influence of anisotropic nano- to micro-topography on in vitro and in vivo osteogenesis. *Nanomedicine*.

[60] Janota C. S., Calero-Cuenca F. J., Gomes E. R. (2020). The role of the cell nucleus in mechanotransduction. *Current Opinion in Cell Biology*.

[61] Gehrig K., Cornell R. B., Ridgway N. D. (2008). Expansion of the nucleoplasmic reticulum requires the coordinated activity of lamins and CTP:pc. *Molecular Biology of the Cell*.

[62] Dalby M. J., Gadegaard N., Tare R. (2007). The control of human mesenchymal cell differentiation using nanoscale symmetry and disorder. *Nature Materials*.

[63] Chaudhary J. K., Rath P. C. (2017). Microgrooved-surface topography enhances cellular division and proliferation of mouse bone marrow-derived mesenchymal stem cells. *PLoS One*.

[64] Li G., Song Y., Shi M., Du Y., Wang W., Zhang Y. (2017). Mechanisms of Cdc42-mediated rat MSC differentiation on micro/nano-textured topography. *Acta Biomaterialia*.

[65] Yang B. J., Xu H. G., Xiao L., Zhang X. L., Wang J., Xu Z. A. (2019). [Regulation of cell deformation induced by RhoA/ROCK signaling pathway in osteogenic differentiation of human mesenchymal stem cells]. *Zhonghua Yixue Zazhi*.

[66] Huang J., Chen Y., Tang C. (2019). The relationship between substrate topography and stem cell differentiation in the musculoskeletal system. *Cellular and Molecular Life Sciences*.

